# Overexpressing p130/E2F4 in mesenchymal stem cells facilitates the repair of injured alveolar epithelial cells in LPS-induced ARDS mice

**DOI:** 10.1186/s13287-019-1169-1

**Published:** 2019-03-06

**Authors:** Xiwen Zhang, Jianxiao Chen, Ming Xue, Yuying Tang, Jingyuan Xu, Ling Liu, Yingzi Huang, Yi Yang, Haibo Qiu, Fengmei Guo

**Affiliations:** Department of Critical Care Medicine, Zhongda Hospital, School of Medicine, Southeast University, No.87 Dingjiaqiao Road, Gulou District, Nanjing, 210009 People’s Republic of China

**Keywords:** Mesenchymal stem cells, Acute respiratory distress syndrome, p130, E2F4, Differentiation into type II alveolar epithelial cells

## Abstract

**Background:**

Low differentiation rates of mesenchymal stem cells (MSCs) limit their therapeutic effects on patients in clinical studies. Our previous study demonstrated that overexpressing p130 or E2F4 affected the multipotential differentiation of MSCs, and the underlying mechanism was attributed to the regulation of the G1 phase. Improving the efficiency of MSC differentiation into epithelial cells is considered to be a new method. Therefore, this study was conducted to evaluate the effects of overexpressing p130 or E2F4 in MSCs on improving re-epithelization in lipopolysaccharide (LPS)-induced ARDS animals.

**Methods:**

Mouse MSCs (mMSCs) stably transfected with p130 and E2F4 were transplanted intratracheally into LPS-induced ARDS mice. After 7 and 14 days, the mice were sacrificed, and the histopathology of the lungs was assessed by haematoxylin-eosin staining and lung injury scoring. Homing and differentiation of mMSCs were analysed by labelling and tracking mMSCs with NIR815 dye and immunofluorescent staining. Surfactant proteins A and C and occludin in the lungs were assessed by western blot. Permeability was evaluated by analysing the protein concentration of BALF using ELISA. Alveolar fluid clearance was assessed by absorbance measurements of BALF. Lung fibrosis was assessed by Masson’s trichrome staining and Ashcroft scoring.

**Results:**

The engraftment of mMSCs overexpressing p130 or E2F4 led to attenuated histopathological impairment of the lung tissue, and the lung injury scores of the LPS+mBM-MSC-p130 and LPS+mBM-MSC-E2F4 groups were also decreased (*p* < 0.05). Overexpression of p130 or E2F4 also increased the retention of mMSCs in the lung (*p* < 0.05), increased differentiation into type II alveolar epithelial cells (*p* < 0.05), and improved alveolar epithelial permeability (*p* < 0.05). Additionally, mMSCs overexpressing p130 or E2F4 inhibited lung fibrosis according to the deposition of collagen and the fibrosis score in the lungs (*p* < 0.05).

**Conclusion:**

Overexpressing p130 or E2F4 in mMSCs could further improve the injured structure and function of epithelial cells in the lungs of ARDS mice as a result of improved differentiation of mMSCs into epithelial cells.

**Electronic supplementary material:**

The online version of this article (10.1186/s13287-019-1169-1) contains supplementary material, which is available to authorized users.

## Background

Mesenchymal stem cells (MSCs), with their property of multipotential differentiation, have been widely used in the treatment of cardiovascular, pulmonary and renal diseases. In a phase 1 clinical trial, allogeneic, bone marrow-derived human MSCs were well tolerated in patients with moderate to severe acute respiratory distress syndrome (ARDS) [1]. Over the past 20 years, studies have shown that MSC transplantation can significantly improve pathological impairment and alleviate inflammation in injured organs. However, low differentiation rates of MSCs limit their therapeutic effects on patients in clinical studies.

ARDS is the major cause of acute respiratory failure in critically ill patients, with an incidence of 26.3 cases/100,000 people [2] and a mortality of more than 40% for moderate to severe ARDS patients despite the use of low-volume and low-pressure ventilation strategies that are aimed at reducing ventilator-induced lung injury [3, 4]. Lung epithelial cell and endothelial cell injury are the basic pathophysiological changes of ARDS. The initial pathophysiological changes of ARDS are characterised by damage of alveolar endothelial and epithelial barriers and accumulation of protein-rich oedema fluid within the interstitium and alveolus [3]. The focus of supportive therapy for ARDS is to further limit lung injury by combining lung-protective ventilation with conservative fluid therapy [5]. Unfortunately, there is currently no pharmacologic therapy for ARDS to reduce mortality [6]. A novel therapeutic method in the clinical approach, which is intravenous delivery of MSCs that interact with injured tissue by releasing a variety of growth factors and differentiate into target cells, seems to be promising for ARDS patients [1, 7]. Our group has been working on MSC treatment of ARDS for many years, and it has been shown that regulation of the canonical and non-canonical Wnt signalling pathways could further improve MSC-mediated protection against epithelial impairment in ARDS mice [8, 9].

The differentiation of cells depends on the efficient control of the cell cycle, in which transcription factors play an important role among different influencing factors. In our previous study, a long-term, stable mMSC line modified with p130/E2F4 was constructed using lentiviral vectors, which regulated the proliferation, migration and differentiation of MSCs. It was also shown that overexpression of p130, a member of the retinoblastoma gene product (pRb) family, or E2F4, a transcriptional repressor in conjunction with p130, in mouse MSCs (mMSCs) improved osteogenesis while inhibiting adipogenesis and chondrogenesis under the regulation of the G1 phase [10]. Improving the efficiency of MSC differentiation into epithelial cells is considered to be a new method. However, the role of p130/E2F4 in the therapeutic effect of MSCs in ARDS remains unexplored in vivo, which may be affected by a more complex environment and regulatory mechanisms that differ from specific and limited culture conditions of differentiation in vitro [10].

Therefore, the aim of this study was to evaluate the effects of overexpressing p130 or E2F4 in MSCs on improving re-epithelization in lipopolysaccharide (LPS)-induced ARDS mice.

## Materials and methods

### Ethics statement

Male wild-type (WT) C57BL/6 mice (Laboratory Animal Center, Shanghai, China), aged 6–8 weeks and weighing 20–25 g, were maintained under specific pathogen-free conditions. All animal experiments performed in this study conformed to the Guide for the Care and Use of Laboratory Animals and were approved by the Institutional Animal Care and Use Committee of Southeast University.

### Mesenchymal stem cell transfection and culture

MSCs derived from the bone marrow of C57BL/6 mice (mBM-MSC) were obtained from Cyagen Biosciences, Inc. (Guangzhou, China). The details of the transfection of mBM-MSCs mediated by lentiviral vectors have been previously described in our work [10]. Briefly, the recombinant lentivirus vectors overexpressing the p130 or E2F4 gene were constructed by using a cytomegalovirus (CMV)-promoter, and an empty CMV-eGFP_IRES was used as an empty vector control. The lentivirus was packaged in 293 T cells (Zoonbio Biotechnology Co., Ltd. Nanjing, China) with the aid of packaging plasmids PDS042-PMD2G and PDS041-PSPAX2, and then, the recombinant lentivirus was used to transfect the mMSCs. mMSCs carrying green fluorescent protein (GFP), namely, normal control mBM-MSC (mBM-MSC-NC) or both p130 or E2F4 with GFP mMSCs (mBM-MSC-p130 or mBM-MSC-E2F4) were harvested after selection using blasticidin (BSD; 6 μg/mL, InvivoGen). Subsequently, mBM-MSC-NC, mBM-MSC-p130 or mBM-MSC-E2F4 were cultured in a 1:1 mixture of Dulbecco’s modified Eagle’s media/nutrient mixture F-12 (DMEM/F12) (Wisent, Inc., St-Bruno, Montreal Quebec, Canada) containing 10% FBS (Wisent, Inc.) and 1% antibiotic-antimycotic solution (streptomycin, penicillin and amphotericin B; Wisent, Inc.) and were incubated at 37 °C in a humidified atmosphere with 5% CO_2_. Cells at passages 6–10 were used for in vivo experiments.

As mentioned in our study [10] before, overexpressing p130 or E2F4 significantly improved osteogenic differentiation while inhibiting adipogenic and chondrogenic differentiation of mMSCs. Moreover, overexpressing p130 or E2F4 significantly improved migration but did not have any effect on proliferation of mMSCs.

### Murine model of lipopolysaccharide-induced acute respiratory distress syndrome

The mice were first anaesthetised with pentobarbital (50 mg/kg) by intra-peritoneal injection and then received an intratracheal (i.t.) administration of LPS (5 mg/kg, *Escherichia coli* serotype 0111: B4; Sigma-Aldrich, St Louis, MO, USA) dissolved in a 20-μL sterile normal saline (NS), which has been described previously [8]. Then, the mice recovered until fully awake in a 100% oxygen chamber, and the control mice received only 0.9% NS instead of LPS.

### Experimental protocol

The mice were randomly divided into six groups as follows: control group, mice received 20-μL phosphate-buffered saline (PBS) intratracheally 4 h after i.t. administration of 0.9% NS; ARDS group, mice received 20-μL PBS intratracheally 4 h after LPS challenge; the LPS+mBM-MSC group received wild-type mBM-MSC (5 × 10^5^ cells resuspended in 20-μL PBS) intratracheally 4 h after LPS challenge; the LPS+mBM-MSC-NC group received mBM-MSC-NC (5 × 10^5^ cells resuspended in 20 μL PBS) intratracheally 4 h after LPS challenge; the LPS+mBM-MSC-p130 group received mBM-MSC-p130 (5 × 10^5^ cells resuspended in 20 μL PBS) intratracheally 4 h after LPS challenge; and the LPS+mBM-MSC-E2F4 group received mBM-MSC-E2F4 (5 × 10^5^ cells resuspended in 20 μL PBS) intratracheally 4 h after LPS challenge. The mice were sacrificed at 7 or 14 days after mMSC injection, and the lung lobes were collected for further analysis.

### Lung histopathology analysis

To examine the severity of lung injury, the right lung lobes (*n* = 3 for each group at each time-point) were collected and fixed in 10% formalin (Shanghai Ling Feng) in PBS. After fixation, the lung lobes were embedded in paraffin and sliced into 5-μm sagittal sections. The sections were stained with a haematoxylin and eosin staining kit (Beyotime Institute of Biotechnology, Haimen, China). The severity of lung injury was analysed by a pathologist based on ten randomly selected high-power fields (400×) in each section according to oedema, alveolar and interstitial inflammation, alveolar and interstitial haemorrhage, atelectasis and necrosis, which was graded on a 0- to 4-point scale (0, no injury; 1, injury in 25% of the field; 2, injury in 50% of the field; 3, injury in 75% of the field; and 4, injury throughout the entire field). The total lung injury score was calculated as the sum of these scores, which has been described previously [8, 11, 12].

### Labelling and tracing of mesenchymal stem cells

Wild-type mBM-MSC, mBM-MSC-NC, mBM-MSC-p130 and mBM-MSC-E2F4 were labelled with CellVue NIR815 dye (eBioscience Inc., San Diego, CA, USA) according to the manufacturer’s instructions. Then, NIR815-labelled cells (5 × 10^5^ cells) were directly administered into the trachea of the mice in different groups according to the protocol. After 7 and 14 days post-transplantation, three mice at each time-point were sacrificed, and ex vivo lungs were imaged using a Maestro in vivo optical imaging system (excitation = 786 nm, emission = 814 nm and 4000 ms exposure time; Calliper Life Sciences, MA, Boston, USA) [8, 13]. The autofluorescence spectra were then unmixed based on their spectral patterns using Maestro 2.4 software (Calliper Life Sciences). The fluorescence intensity of the lungs was measured by placing the regions of interest (ROIs) on the lungs, and the signals were analysed based on the total fluorescence counts of the ROIs.

### Immunofluorescent staining

To analyse the recruitment of mMSCs into the lungs and their differentiation in vivo, immunofluorescent staining was also performed as previously described [14]. Briefly, the left lung lobes (*n* = 3 per group at each time-point) were snap frozen in liquid nitrogen and then stored at − 80 °C until use. After being embedded in optimal cutting temperature (OCT) compound (Sakura Finetek USA, Inc., Torrance, CA, USA), the tissues were cut into 5-μm-thick sections. Then, the slides were fixed in acetone at 4 °C for 15 min, ruptured by 0.3% Triton X-100 and then blocked with 3% bovine serum albumin (BSA; Roche, Ltd., Basel, Switzerland) for 30 min at room temperature. Following incubation overnight at 4 °C, the slides were stained with GFP primary antibody (1:100 dilution, Abcam, Cambridge, MA, USA) alone or with surfactant protein C (SP-C) primary antibodies (1:100 dilution, Santa Cruz Biotechnology, Paso Robles, CA, USA) at the same volume. Then, these slides were incubated with secondary FITC-labelled goat anti-rabbit IgG (H+L) (1:1000 dilution, Beyotime) and goat anti-rabbit Alexa Fluor® 647 antibodies (1:200 dilution, Abcam) in 2% BSA for 1 h at 37 °C in the absence of light. The nuclei were stained with 4,6-diamidino-2-phenylindole (DAPI; Sigma-Aldrich) for 5 min. Images were acquired by fluorescence microscopy (Olympus, Tokyo, Japan). The retention of transplanted mMSCs was quantified based on the overlap of DAPI- and GFP-positive mMSCs in randomly selected fields by Image-Pro Plus 6.0 (Media Cybernetics, Bethesda, MD, USA), and the differentiation of transplanted mMSCs was analysed by the overlap of DAPI-, GFP- and SP-C-positive mMSCs.

### Protein expression of SP-A, SP-C and occludin in the lung

To analyse the expression of SP-A, SP-C and occludin in the lungs after transplantation, total protein lysates were extracted by RIPA lysis buffer (Beyotime) from left lung lobes (*n* = 3 per group at each time-point) and then quantified by a BCA protein assay kit (Beyotime) as previously described [9]. The proteins were separated by 8% or 10% sodium dodecyl sulfate-polyacrylamide gel electrophoresis (SDS-PAGE) (Beyotime) and electro-transferred onto PVDF membranes (Millipore, Bedford, MA, USA). After blocking in tris-buffered saline (TBS; pH 7.4; Biosharp Biotechnology, Hefei, China) containing 0.1% Tween-20 (TBST; Shanghai Chemical Reagent Company of China Pharmaceutical Group, Shanghai, China) and 5% BSA for 1 h at room temperature, the membranes were incubated at 4 °C overnight with primary antibodies against SP-A (1:1000 dilution, Abcam), SP-C (1:100 dilution, Abcam), β-actin (1:3000 dilution, Hangzhou HuaAn Biotechnology, Co., Ltd., China) or occludin (1:1000 dilution; Abcam). Subsequently, the blots were washed with TBST and incubated with goat anti-rabbit or goat anti-mouse IgG conjugated with horseradish peroxidase (1:5000 dilution; Zoonbio Biotechnology, Nanjing, China) for 1 h at room temperature. Then, immunoreactive complexes were detected by Pierce ECL western blotting substrate (Thermo Fisher Scientific, Inc., Waltham, MA, USA), and immunoreactive bands were obtained using a chemiluminescence imaging system (Bioshine ChemiQ 4800 mini; Ouxiang, Shanghai, China). Finally, intensity of those bands was analysed by ImageJ software (NIH, USA).

### Protein concentration in bronchoalveolar lavage fluid

Bronchoalveolar lavage fluid (BALF) was collected by flushing 1-mL ice-cold PBS back and forth three times through a tracheal cannula. After centrifugation at 800 × *g* for 10 min, the total protein and albumin concentrations in the BALF were measured as a marker of epithelial permeability by ELISA kits (Cusabio Biotech, Wuhan, China) as previously described [8].

### Evaluation of lung oedema

Lung oedema was evaluated using the ratio of lung wet weight to body weight (LWW/BW) that was measured as previously described [15]. Briefly, the whole lung was removed and cleared of all extrapulmonary tissues, and the LWW/BW was calculated based on the values of the lung wet weight and the body weight (mg/g).

### Evaluation of alveolar fluid clearance

To evaluate alveolar fluid clearance (AFC) of ARDS mice in each group, 80-μL PBS with 5% BSA was administered intratracheally into anaesthetized mice. One hour later, the alveolar fluid was aspirated, and the absorbance was measured using a spectrophotometer. The AFC was calculated using the following formula: AFC (%/hour) = [(Cf-Ci)/Cf] × 100%, where Ci is the initial absorbance value before administration, and Cf is the final absorbance value after aspiration [16, 17].

### Masson’s trichrome staining and fibrosis scoring

The lung sections were stained sequentially with Weigert’s iron haematoxylin solution, Biebrich scarlet-acid fuchsin solution and aniline blue solution, and a blue signal indicated positive staining for collagen. The criteria of Ashcroft were used [18] to assess lung fibrosis, which was quantified based on the findings in ten randomly selected high-power fields (400×) for each slide by histopathologists blinded to the protocol.

### Statistical analysis

The data are presented as the means ± standard deviation (SD). Statistical analyses were performed using SPSS 22.0 (SPSS Inc., Chicago, IL, USA) and GraphPad Prism 6 (GraphPad Software, La Jolla California USA). Comparisons among multiple groups were performed by one-way ANOVA followed by Bonferroni’s post hoc test if the data were normally distributed. A *p* value < 0.05 was considered statistically significant.

## Results

### Mesenchymal stem cells overexpressing p130 or E2F4 improved the pulmonary histopathology of lipopolysaccharide-induced ARDS mice

After LPS-induced lung injury, alveolar wall thickening, alveolar and interstitial inflammatory cell infiltration, haemorrhage, alveolar exudate and oedema were observed in the lung tissues of ARDS group mice (Fig. 1b), and the Smith score for quantifying lung injury was also increased significantly (*p* < 0.05, Fig. 1g) in the ARDS group. However, compared to the ARDS group, histopathologic characteristics and the Smith score were alleviated at 7 and 14 days in the LPS+mBM-MSC and LPS+mBM-MSC-NC groups (*p* < 0.05, Fig. 1c, d, and g). The effects were greater in the LPS+mBM-MSC-p130 group and the LPS+mBM-MSC-E2F4 group than in the LPS+mBM-MSC-NC group (*p* < 0.05) (Fig. 1d–g).

**Fig. 1:** The effect of mMSCs overexpressing p130 or E2F4 on the histopathology of LPS-induced lung injury in mice. **a**–**f** Representative histopathological images of the lung tissues from mice of all the experimental groups at 7 and 14 days after LPS challenge (HE staining, × 200). Alveolar wall thickening was marked as red triangle. Inflammatory cell infiltration was marked as yellow arrow, and haemorrhage was marked as green arrow. **g** Lung injury score (Smith score) of the lung tissues from mice of all the experimental groups at 7 and 14 days after LPS challenge (*n* = 3 at each time-point for each group; *p < 0.05 compared with the control group; #*p* < 0.05 compared with the ARDS group; δ*p* < 0.05 compared with the LPS+MSC-NC group). ARDS acute respiratory distress syndrome, mMSCs mouse mesenchymal stem cells, NC normal control

### Overexpression of p130 or E2F4 increased the retention of mesenchymal stem cells in the lung after lipopolysaccharide challenge

To track intrapulmonary mMSCs, ex vivo NIR imaging and immunofluorescence staining were performed on the lungs at 7 and 14 days after mMSC administration. Fluorescent counts of ROIs in the LPS+mBM-MSC-p130 and LPS+mBM-MSC-E2F4 groups were greater than those in the LPS+mBM-MSC-NC group at 7 days after mMSC administration (*p* < 0.05). Although there were no significant differences among the groups at 14 days (*p* > 0.05), there was still an upward trend of the fluorescent counts in the LPS+mBM-MSC-p130 and LPS+mBM-MSC-E2F4 groups (Fig. 2a, b).

**Fig. 2:** The effect of overexpressing p130 or E2F4 on the retention of mMSCs in the lungs after LPS challenge (NIR imaging). **a** Representative ex vivo NIR images of injured lungs from mice at 7 and 14 days after mMSC administration. **b** Fluorescent counts from ex vivo NIR imaging of injured lungs from mice at 7 and 14 days after mMSC administration (*n* = 3; *p < 0.05 compared with the LPS+MSC-NC group). mMSCs mouse mesenchymal stem cells, NIR near-infrared fluorescent

For the immunofluorescence staining, the results were consistent with the results of NIR imaging and showed that the number of GFP-positive cells was significantly higher in injured lung tissues of the LPS+mBM-MSC-p130 and LPS+mBM-MSC-E2F4 groups than in those of the LPS+mBM-MSC-NC group at both 7 and 14 days after mMSC administration (Fig. 3a, b).

**Fig. 3:** The effect of overexpressing p130 or E2F4 on the retention of mMSCs in the lungs after LPS challenge (immunofluorescent imaging). **a** Representative immunofluorescent staining images of the lung tissues from mice at 7 and 14 days after mMSC administration. mMSC engraftment in the lung tissues is shown as GFP-positive cells (green). Nuclei of cells were stained with DAPI (blue). Double-stained cells with both GFP and DAPI were light green. Representative photographs are shown from three mouse lungs at 7 and 14 days after mMSC administration. All microphotographs were acquired at × 200 magnification (scale bar = 50 μm). **b** Fluorescent counts in injured lungs from mice at 7 and 14 days after mMSC administration. Overlapping fluorescence of DAPI and GFP was counted in randomly selected fields (count/field) (*n* = 3; *p < 0.05 compared with the LPS+MSC-NC group). mMSCs mouse mesenchymal stem cells, GFP green fluorescent protein

### Overexpression of p130 or E2F4 promoted the differentiation of mesenchymal stem cells into type II alveolar epithelial cells in vivo

To assess the differentiation of mMSCs into type II alveolar epithelial cells (AT II) in vivo, immunofluorescence staining of SP-C and the protein expression of SP-A and SP-C in mMSC-grafted lungs were analysed at 7 and 14 days after mMSC administration. Co-localization of SP-C (red) and MSCs (green) in the lung tissue, which appeared white, was observed in the LPS+mBM-MSC-NC, LPS+mBM-MSC-p130 and LPS+mBM-MSC-E2F4 groups; however, the mBM-MSC-p130 and mBM-MSC-E2F4 treatments led to a greater differentiation efficiency of the mMSCs into AT II than the mBM-MSC-NC treatment at both 7 and 14 days after mMSC transplantation (Fig. 3a, b).

The total protein expression of SP-A and SP-C in lung tissues at 7 and 14 days after mMSC administration was evaluated by western blot analysis. Both SP-A and SP-C were upregulated in the LPS+mBM-MSC and LPS+mBM-MSC-NC groups compared with the ARDS group at 7 days (*p* < 0.05). Compared to the LPS+mBM-MSC-NC group, SP-A and SP-C protein expression levels increased significantly in the LPS+mBM-MSC-p130 and LPS+mBM-MSC-E2F4 groups at 7 days (*p* < 0.05) (Fig. 4c). However, at 14 days after mMSC administration, the SP-A protein expression level in the LPS+mBM-MSC-p130 and LPS+mBM-MSC-E2F4 groups but not in the LPS+mBM-MSC and LPS+mBM-MSC-NC groups increased significantly compared to that in the ARDS group (*p* < 0.05), while the SP-A protein expression level in the LPS+mBM-MSC-p130 and LPS+mBM-MSC-E2F4 groups was increased significantly compared to that in the LPS+mBM-MSC-NC group (*p* < 0.05). The SP-C protein expression level increased significantly in the LPS+mBM-MSC and LPS+mBM-MSC-NC groups compared with that in the ARDS group (*p* < 0.05). Moreover, SP-C protein expression was also upregulated significantly in the LPS+mBM-MSC-p130 and LPS+mBM-MSC-E2F4 groups compared to that in the LPS+mBM-MSC-NC group (*p* < 0.05) (Fig. 4c, relative intensity of each band on the representative image was shown in Additional file 1).

**Fig. 4:** The effect of overexpressing p130 or E2F4 on the differentiation of mMSCs into AT II in vivo. **a** Representative immunofluorescent staining images of the injured lungs from mice at 7 and 14 days after mMSC administration. mMSC engraftment in the lung tissues (GFP-positive cells) appears green, the specific marker of AT II (SP-C) appears red and the nuclei of cells that were stained with DAPI appear blue. Double-stained cells with both GFP and DAPI appear light green. The co-localization of green, red and blue appears white. Representative photographs are shown from three mouse lungs at 7 and 14 days after mMSC administration. All microphotographs were acquired at × 200 magnification (scale bar = 50 μm). **b** Fluorescent counts in the injured lungs from mice at 7 and 14 days after mMSC administration. Overlapping fluorescence of DAPI, GFP and SP-C was counted in randomly selected fields (count/field) (*n* = 3; *p < 0.05 compared with the LPS+MSC-NC group). **c** The protein expression of SP-A and SP-C in the lung tissue at 7 and 14 days after mMSC administration was evaluated by western blot analysis (*n* = 3, *p < 0.05 compared with the control group; #*p* < 0.05 compared with the ARDS group; δ*p* < 0.05 compared with the LPS+MSC-NC group). ARDS acute respiratory distress syndrome, AT II type II alveolar epithelial cells, mMSCs mouse mesenchymal stem cells, GFP green fluorescent protein, SP-A surfactant protein A, SP-C surfactant protein C

### Overexpression of p130 or E2F4 in mesenchymal stem cells improved the function of type II alveolar epithelial cells and reduced the high permeability of ARDS

The LWW/BW was calculated to evaluate lung oedema. The LWW/BW was significantly reduced in the LPS+mBM-MSC and LPS+mBM-MSC-NC groups compared with that in the ARDS group at 7 and 14 days (*p* < 0.05). At 14 days, the LWW/BW also decreased significantly in the LPS+mBM-MSC-p130 and LPS+mBM-MSC-E2F4 groups compared to that in the LPS+mBM-MSC-NC group (Fig. 5a).

**Fig. 5:** The effect of mMSCs overexpressing p130 or E2F4 on the permeability of LPS-induced lungs in mice. **a** Lung oedema was analysed by LWW/BW. The results are shown for samples of all the experimental groups at 7 and 14 days after LPS exposure (*n* = 3, *p < 0.05 compared with the control group; #*p* < 0.05 compared with the ARDS group; δ*p* < 0.05 compared with the LPS+MSC-NC group). **b** Total protein and **c** albumin concentrations in bronchoalveolar lavage fluid were analysed by a mouse-specific ELISA kit to evaluate the epithelial permeability of the lung (*n* = 3, *p < 0.05 compared with the control group; #*p* < 0.05 compared with the ARDS group; δ*p* < 0.05 compared with the LPS+MSC-NC group). **d** Expression of the occludin protein in the lungs of all the experimental groups at 7 and 14 days after mMSC administration was evaluated by western blot analysis (*n* = 3, *p < 0.05 compared with the control group; #*p* < 0.05 compared with the ARDS group; δ*p* < 0.05 compared with the LPS+MSC-NC group). **e** Alveolar fluid clearance was measured at 7 and 14 days after mMSC administration (*n* = 3, *p < 0.05 compared with the control group; #*p* < 0.05 compared with the ARDS group; δ*p* < 0.05 compared with the LPS+MSC-NC group). ALB albumin, ARDS acute respiratory distress syndrome, ELISA enzyme-linked immunosorbent assay, LWW/BW lung wet weight/body weight, mMSCs mouse mesenchymal stem cells, NC normal control, TP total protein

To evaluate whether mMSCs overexpressing p130 or E2F4 could make a difference in the epithelial permeability of the lung, total protein and albumin concentrations in the BALF were measured by mouse-specific ELISAs. The total protein and albumin concentrations were significantly reduced in the LPS+mBM-MSC and LPS+mBM-MSC-NC groups compared with those in the ARDS group at 7 days (*p* < 0.05), while no difference was observed at 14 days. Significant decreases in the total protein and albumin concentrations were also observed in the LPS+mBM-MSC-p130 and LPS+mBM-MSC-E2F4 groups compared with the LPS+mBM-MSC-NC group at 7 and 14 days (*p* < 0.05) (Fig. 5b, c).

Additionally, occludin protein expression, which is a marker of tight junctions of pulmonary epithelial cells, was evaluated in lung tissue at 7 and 14 days after mMSC administration by western blot analysis. The occludin protein expression level increased significantly in the LPS+mBM-MSC and LPS+mBM-MSC-NC groups compared with that in the ARDS group (*p* < 0.05). A significant increase was also observed in the LPS+mBM-MSC-p130 and LPS+mBM-MSC-E2F4 groups compared to the ARDS group (*p* < 0.05), and the increase was much greater than that in the LPS+mBM-MSC-NC group (*p* < 0.05) (Fig. 5d, relative intensity of each band on the representative image was shown in Additional file 1).

In addition, to investigate the ability of AT II to clear lung water, the AFC was measured at 7 and 14 days after mMSC administration. The results showed that there was a significant increase in the AFC in the LPS+mBM-MSC and LPS+mBM-MSC-NC groups compared to that in the ARDS group at both 7 and 14 days (*p* < 0.05). Although there was only an upward trend of the AFC in the LPS+mBM-MSC-p130 and LPS+mBM-MSC-E2F4 groups compared to that in the LPS+mBM-MSC-NC group at 7 days, a significant increase was observed at 14 d (*p* < 0.05) (Fig. 5e).

### Mesenchymal stem cells overexpressing p130 or E2F4 inhibited lung fibrosis in ARDS mice

To assess lung fibrosis, collagen deposition (which was stained as blue) in the lung tissue at 14 days after LPS challenge was analysed by Masson’s trichrome staining and was markedly increased in the ARDS group compared with that in the control group (*p* < 0.05). The lung fibrosis score decreased significantly in the LPS+mBM-MSC and LPS+mBM-MSC-NC groups compared to that in the ARDS group (*p* < 0.05). Reduced deposition of collagen was observed after intervention with either mBM-MSC-p130 or mBM-MSC-E2F4 compared with the ARDS group (*p* < 0.05), but the decreased deposition of collagen observed in the LPS+mBM-MSC-p130 and LPS+mBM-MSC-E2F4 groups was more significant than that observed in the LPS+mBM-MSC-NC group (*p* < 0.05) (Fig. 6a, b).

**Fig. 6:** The effect of mMSCs overexpressing p130 or E2F4 on lung fibrosis in ARDS mice. **a** Lung fibrosis was evaluated by Masson’s trichrome staining at 14 days after LPS exposure (× 200). A blue signal indicated positive staining for collagen, and a red signal represented muscle fibrosis and cellulose. **b** The quantification of lung fibrosis is shown as an Ashcroft score (*n* = 10, *p < 0.05 compared with the control group; #*p* < 0.05 compared with the ARDS group; δ*p* < 0.05 compared with the LPS+MSC-NC group)

## Discussion

In recent decades, there has been no significant breakthrough in the treatment of ARDS using MSCs in clinical experiments, mainly because of the retention and directional differentiation of MSCs in the injured lungs. In this study, mMSCs overexpressing p130 or E2F4 were constructed in vitro and transplanted intratracheally into LPS-induced ARDS mice for the first time. It was found that (1) mMSCs overexpressing p130 or E2F4 further attenuated pathological damage in ARDS mice after transplantation; (2) mMSCs overexpressing p130 or E2F4 further attenuated the injuries of AT II in ARDS mice, further improving not only the structure but also their functions; (3) mMSCs overexpressing p130 or E2F4 further increased the retention of MSCs in ARDS mice after transplantation; and (4) mMSCs overexpressing p130 or E2F4 decreased pulmonary fibrosis in ARDS mice.

Intravenous delivery of MSCs, which is a novel therapeutic method for clinical approaches, seems to be promising for ARDS patients [7, 19]. Previous studies confirmed that MSC transplantation significantly attenuated pathological damage in ARDS mice [8, 12, 15, 20], which was also observed in this study. However, our study focused on the nature of MSCs with respect to their basic characteristics of cell differentiation to demonstrate the role of regulating the cell cycle on MSC directional differentiation in vivo. Our previous study [10] showed that overexpressing p130 or E2F4 affected the differentiation of MSCs in vitro by G1 phase regulation, which is the primary node of cell differentiation. Therefore, the mechanism by which MSCs improve pathological damage in ARDS mice may be associated with the directional differentiation of MSCs after transplantation.

To further study the directional differentiation of MSCs in the lung, SP-C was used as the main marker of AT II to verify the efficiency of MSC differentiation after transplantation, and the function of differentiated epithelial cells was analysed by an alveolar fluid clearance test. This may also be the first study to show that overexpressing p130 or E2F4 in MSCs could significantly increase their differentiation into AT II and improve the function of epithelial cells in ARDS mice. p130, which is a member of the retinoblastoma gene product (pRb) family, controls the exit from the G1 phase [21]. It can also form a repressor complex with the transcription factor E2F4, which is a transcriptional repressor whose activity is critical for the engagement and maintenance of cell cycle arrest in G0/G1 in conjunction with members of the retinoblastoma (Rb) family. It has been previously shown that the p130/E2F4 complex is associated with embryonic stem cell differentiation [22]. Our previous study also showed that cell cycle regulation may be involved in p130-/E2F4-mediated changes in the multipotential abilities of bone marrow-derived mMSCs [10]. Therefore, it can be speculated that the possible mechanism of the improved differentiation of MSCs into AT II could depend on a prolonged G1 phase, which is associated with the overexpression of p130 or E2F4 according to our results.

In addition to directional differentiation, MSC retention in the lungs remains the main obstruction to MSCs therapy. It has been previously shown that less than 8% of MSCs remained at 3 days after MSC delivery in LPS-challenged mouse lungs [23]. In our study, it was shown that overexpressing p130 or E2F4 significantly improved MSC retention at 7 days but not at 14 days after transplantation, as suggested by the NIR imaging results. However, an upward trend for their retention was also observed by immunofluorescence staining. However, there is currently still no similar research to corroborate this result, and further studies need to be conducted to elucidate the mechanism.

Pulmonary fibrosis may be a major complication after MSC transplantation in ARDS. Because of the multidirectional differentiation potential of MSCs, MSCs cannot only differentiate into alveolar epithelial cells but also differentiate into pulmonary fibroblasts and myofibroblasts, secreting collagen and resulting in pulmonary fibrosis [24, 25]. A previous study has shown that irradiation-induced pulmonary fibrotic tissue contains proliferating cells of bone marrow origin [26]. In this study, Masson’s trichrome staining was used to analyse pulmonary fibrosis after mMSC transplantation. Surprisingly, it was shown that mMSCs overexpressing p130 or E2F4 decreased pulmonary fibrosis in ARDS mice, which provided a good foundation for the transplantation of mMSCs overexpressing p130 or E2F4.

There were two limitations in this study. First, the LPS-induced ARDS model is the most common model, but it does not represent different types of causes of ARDS. Second, because the role of epithelial cells in ARDS was a substantial focus of this study, indicators associated with endothelial cells in ARDS were not analysed and were not a focus of this study.

## Conclusions

In conclusion, it was shown that overexpressing p130 or E2F4 increased the retention of mMSCs in the lungs of ARDS mice and promoted the differentiation of mMSCs into AT II, thereby improving lung permeability and pulmonary fibrosis, reducing pulmonary oedema and further contributing to an improved therapeutic effect of mMSCs on ARDS mice. This study provided a new research focus for our follow-up study of the MSC-based treatment of ARDS.

## Additional file

Additional file 1: Relative intensity of each band on the representative image of western blot. The relative intensity of bands on the representative images of SP-A, SP-C and occludin in Western blot was shown in Additional file 1 (XLSX 9 kb)

## Abbreviations

AFC: Alveolar fluid clearance
ARDS: Acute respiratory distress syndrome
AT II: Type II alveolar epithelial cells
BALF: Bronchoalveolar lavage fluid
BSA: Bovine serum albumin
DAPI: 4,6-Diamidino-2-phenylindole
DMEM/F12: Dulbecco’s modified Eagle’s media/nutrient mixture F-12
ELISA: Enzyme-linked immunosorbent assay
GFP: Green fluorescent protein
LPS: Lipopolysaccharide
LWW/BW: Lung wet weight/body weight
mMSCs: Mouse mesenchymal stem cells
MSC-E2F4: Mesenchymal stem cells overexpressing E2F4
MSC-NC: Mesenchymal stem cells carrying green fluorescent protein (normal control)
MSC-p130: Mesenchymal stem cells overexpressing p130
MSCs: Mesenchymal stem cells
NIR: Near-infrared fluorescent
NS: Normal saline
OCT: Optimal cutting temperature
PBS: Phosphate-buffered saline
pRb: Retinoblastoma gene product
Rb: Retinoblastoma
RIPA: Radioimmunoprecipitation assay buffer
SD: Standard deviation
SDS-PAGE: Sodium dodecyl sulfate-polyacrylamide gel electrophoresis
SP-A: Surfactant protein A
SP-C: Surfactant protein C
TBS: Tris-buffered saline
TBST: Tris-buffered saline with Tween-20
